RETRACTED

# Meta-analysis of the efficacy of pancreatoduodenectomy with extended lymphadenectomy in the treatment of pancreatic cancer

**DOI:** 10.1186/1477-7819-11-311

**Published:** 2013-12-10

**Authors:** Xinbao Xu, Hui Zhang, Ping Zhou, Lei Chen

**Affiliations:** 1 Department of Hepatobiliary Surgery, Airforce General Hospital of Chinese People's Liberation Army, Beijing 100142, China; 2 Department of Radiotherapy, Airforce General Hospital of Chinese People's Liberation Army, Beijing 100142, China; 3 Department of Hepatobiliary Surgery, Peking University People’s Hospital, Beijing 100044, China

**Keywords:** Pancreatic cancer, Pancreatoduodenectomy with extended lymphadenectomy, Standard pancreatoduodenectomy, Meta-analysis

## Abstract

**Background:**

The purpose of this meta-analysis is to compare the efficacy of pancreatoduodenectomy (PD) with extended lymphadenectomy (PD/ELND) versus standard PD in the treatment of pancreatic cancer, with the hope of providing evidence for clinical practice.

**Methods:**

The retrieval of relevant literature published before September 2012 was carried out on PubMed, Medline, Embase, and Cochrane Central Register of Controlled Trials (CENTRAL) by computer. Information was extracted according to Cochrane systematic review methods, and analyzed using software Stata 11.0.

**Results:**

Five prospective randomized controlled trials (RCTs) were included in this meta-analysis of 555 cases (278 in the PD/ELND group and 277 in the standard PD group). The PD/ELND group showed a significantly lower 3-year survival rate (relative risk (RR) = 1.46, 95% confidence interval (CI) 1.03 to approximately 2.06, *P* = 0.034), prolonged operative time (weighted mean difference WMD = −1.03, 95% CI −1.96 to approximately −0.10, *P* = 0.029) and higher incidence of postoperative complications (RR = 0.56, 95% CI 0.42 to approximately 0.77, *P* = 0.000) by comparing with standard PD group. Besides, no significant difference was observed in the 1-year survival rate (RR = 0.87, 95% CI 0.60 to approximately 1.25, *P* = 0.69), 5-year survival rate (RR = 1.04, 95% CI 0.68 to approximately 1.58, *P* = 0.854), postoperative mortality (RR = 1.14, 95% CI 0.43 to approximately 3.00, *P* = 0.789), length of stay (WMD = −0.32, 95% CI −2.57 to approximately 1.94 , *P* = 0.784) and the amount of blood transfusions (WMD = −0.14, 95% CI −0.36 to approximately 0.08, *P* = 0.213).

**Conclusions:**

PD/ELND does not have an advantage over standard PD in the survival rate for patients with pancreatic cancer, but does increase operative time and incidences of postoperative complications.

## Background

Pancreatic cancer case about 20 million deaths worldwide each year with an increasing incidence. Now, pancreatic cancer has become the fourth leading cause of death among cancers, and is one of the common gastrointestinal malignancies. It possesses some characteristics, such as fast progress, high degree of malignancy and early metastasis, which eventually bring poor prognosis for patients with a 5-year survival rate of only l% to 3% [1,2]. Currently, surgery is still the most basic means for treating pancreatic cancer, also the only method of hoping for curative treatment. Since the first successful implementation of surgery in 1935 by Whipple, pancreatoduodenectomy (PD) has been the standard operation for pancreatic cancer [3]. As pancreatic cancer spreads to regional lymph nodes and even to the pancreas plexus along the perineurium, efforts to improve the surgical method have been based on conventional PD and variations of extended PD, such as pancreatoduodenectomy with extended lymphadenectomy (PD/ELND) [4].

RETRACTED

However, the use of PD/ELND is controversial at home and abroad. In 1973, Fortner [5] suggested that regional resection should include the pancreas and the immediate area of lymphatic drainage. But it was not widely accepted because there was no solid evidence to support this technique. However, Ishikawa [6] proposed an improved 3-year survival rate with an extended lymphadenectomy in 1988. Subsequently, several studies were carried out to explore the efficacy of extended surgery with conflicting conclusions. For example, Tadao Manabe *et al*. showed that the survival rates in patients treated with radical operation were significantly higher than in patients with nonradical operation [7], and Naganuma *et al*. showed that extended resection in Japan can improve the curative resection and actuarial survival rate compared with standard resection [8]. In a study by Satake *et al*., however, no significant difference was observed in the overall postoperative cumulative survival rates between the standard and extended operation [9].

Meta-analysis, as a statistical analysis method, can quantitatively pool a number of independent clinical studies and provide some information to resolve the controversial and uncertain questions. Therefore, we collected relevant literature and performed a meta-analysis to systematically assess the clinical efficacy of PD/ELND and standard PD and to provide evidences for the clinical applications of PD/ELND.

## Methods

Literatures that compared the efficacy of PD/ELND and standard PD in the treatment of pancreatic cancer was retrieved through searches of PubMed, Medline, Embase and Cochrane Central Register of Controlled Trials (CENTRAL) by computer, and supplemented by manual searches and reference backtracking. The deadline was set for September 2012. The following words or terms were adopted as keywords or key terms: pancreatic cancer, pancreatic adenocarcinoma, pancreatoduodenectomy, pancreatoduodenectomy with extended lymphadenectomy, *etcetera*.

RETRACTED

### Inclusion and exclusion criteria

The inclusion and exclusion criteria in this meta-analysis were as follows: (1) English literatures published abroad were included except for non-original literatures and review literatures; (2) the objects of study should be patients with pancreatic cancer(approved by ethics committee of the Airforce General Hospital of Chinese People's Liberation Army; (3) prospective randomized controlled trials (RCTs) were included whereas retrospective studies, non-RCTs and case reports were excluded; (4) PD/ELND was required for patients to be assigned the test group whereas standard PD was used to assign patients to the control group; (5) complete data were available with a specific number of cases; (6) diagnostic criteria and therapeutic evaluation indicators were clearly described; and (7) at least one of the following indicators was included (operative time, postoperative hospital stay, amount of blood transfusions, incidence of postoperative complications, postoperative mortality, postoperative 1-, 3- and 5-year survival rate).

### Data extraction

Two researchers independently assessed literatures for the following aspects: (1) general information (first author, publication year, source, and publication date); (2) study design; (3) number of cases, demographic characteristics, and treatment outcomes; and (4) conclusions.

### Statistical analysis

Meta-analysis was performed using software Stata 11.0 (StataCorp LP, Texas,USA).

The standardized weighted mean difference (WMD) with corresponding 95% confidence interval (CI) was calculated for continuous data, while relative risk (RR) with 95% CI was determined for dichotomous data. The significance level was set as 0.05. Heterogeneity between studies was detected with a Chi-square test before pooling data, and the quantity of heterogeneity was measured by using the I^2^ statistic. A fixed effects model was used if *P* >0.05 according to test, while a random effects model was adopted if *P* ≤0.05.

Additionally, to assess the influence of the trial quality on our meta-analysis, we performed the sensitivity analysis by including only the trials that included a majority of adult patients with pancreatic cancer.

## Results

### Basic information

After searching the studies by the keywords or key terms, 90 relevant literatures were obtained after a preliminary screening. Then, these literatures were further screened according to inclusion and exclusion criteria. Finally, five studies, Pedrazzoli *et al*. [10], Farnell *et al*. [11], Yeo *et al*. [12], Riall *et al*. [13] and Nimura *et al*. [14] were included in this meta-analysis. All five studies were prospective RCTs with a total of 555 cases: 278 in the PD/ELND group and 277 in the standard PD group. They were published during the period 1998 to 2012. Basic information such as authors, research time, country, age of patients, sex ratio, number of cases in test group, number of cases in control group and indicators is shown in Table 1.

RETRACTED

**Table 1:** Basic information for studies included in the meta-analysis

**Authors**	**Research time**	**Country**	**Average age (PD/ELND versus PD)**	**Male/Female (PD/ELND versus PD)**	**Number of cases (PD/ELND versus PD)**	**Indicators**
Pedrazzoli *et al*. [10]	3/1991 to 3/1994	Italy	59.2/62	25/16	41/40	operative time, postoperative hospital stay, amount of blood transfusions, incidence of postoperative complications, mortality, 4-year survival rate
				27/13		
Farnell *et al*. [11]	5/1997 to 7/2003	U.S.	67/66	18/21	39/40	operative time, postoperative hospital stay, incidence of postoperative complications, mortality, 1-, 3-, and 5-year survival rate,
				20/20		
Yeo *et al*. [12,13]	4/1996 to 6/2001	U.S.	65.2/66.2	76/72	148/146	operative time, postoperative hospital stay, amount of blood transfusions, incidence of postoperative complications, mortality, 1-, 3-, and 5-year survival rate
				85/61		
Nimura *et al*. [14]	2000.3 to 2003.5	Japan	61/62	25/26	51/50	operative time, postoperative hospital stay, amount of blood transfusions, incidence of postoperative complications, mortality, 1-, 3-, and 5-year survival rate
				25/25		

PD, pancreatoduodenectomy; PD/ELDN, pancreatoduodenectomy with extended lymphadenectomy.

### Efficacy evaluation of pancreatoduodenectomy with extended lymphadenectomy in treatment of pancreatic cancer

#### Postoperative 1-year survival rate

A total of four studies [11-14] described the 1-year survival rate for patients with pancreatic cancer. As between-study heterogeneity was not observed (*P* = 0.117, I^2^ = 53.3%), a fixed effects model was used for analysis. No significant difference was identified in 1-year survival rate between the PD/ELND group and the standard PD group according to the analysis result (RR = 0.87, 95% CI 0.60 to approximately 1.25, *P* = 0.69, Figure 1).

**Figure 1:** **Forest plot for the 1-year survival rate between the pancreatoduodenectomy with extended lymphadenectomy (PD/ELND) group and the standard pancreatoduodenectomy (PD) group.** On the left, the name of the first author of the study is followed by the publication year. The size of the black box corresponding to each study is proportional to the sample size, and the horizontal line shows the corresponding 95% CI of the relative risk (RR) displayed on the right.

RETRACTED

#### Postoperative 3-year survival rate

In these five published articles, four studies [11-14] reported the 3-year survival rate of the patients with PD/ELND and PD. Due to a lack of between-study heterogeneity (*P* = 0.117, I^2^ = 53.4%), a fixed effects model was used for further analysis. We found that the 3-year survival rate of the standard PD group was significantly higher than that of the PD/ELND group (RR = 1.46, 95% CI 1.03 to approximately 2.06, *P* = 0.034, Figure 2).

**Figure 2:** **Forest plot for the 3-year survival rate between the pancreatoduodenectomy with extended lymphadenectomy (PD/ELND) group and the standard pancreatoduodenectomy (PD) group.** The size of the black box corresponding to each study is proportional to the sample size, and the horizontal line shows the corresponding 95% CI of the relative risk (RR) displayed on the right.

#### Postoperative 5-year survival rate

The 5-year survival rate was also reported in four studies [11-14]. Because between-study heterogeneity was still absent in the result (*P* = 0.098, I^2^ = 56.9%), a fixed effects model was applied in this meta-analysis. No obvious difference was observed in 5-year survival rate between the PD/ELND group and the standard PD group (RR = 1.04, 95% CI 0.68 to approximately 1.58, *P* = 0.854, Figure 3).

**Figure 3:** **Forest plot for the 5-year survival rate between the pancreatoduodenectomy with extended lymphadenectomy (PD/ELND) group and the standard pancreatoduodenectomy (PD) group.** The size of the black box corresponding to each study is proportional to the sample size, and the horizontal line shows the corresponding 95% CI of the relative risk (RR) displayed on the right.

#### Incidence of postoperative complications

In all five studies [10-14], the incidence of postoperative complications of patients with pancreatic cancer was detected. The between-study heterogeneity was not observed (*P* = 0.523, I^2^ = 0.0%); therefore a fixed effects model was used for analysis. According to the meta-analysis results (RR = 0.56, 95% CI 0.42 to approximately 0.77, *P* = 0.000, Figure 4), the incidence of postoperative complications in PD/ELND group was significantly higher than that in standard PD group.

**Figure 4:** **Forest plot for the incidence of postoperative complications between the pancreatoduodenectomy with extended lymphadenectomy (PD/ELND) group and the standard pancreatoduodenectomy (PD) group.** The size of the black box corresponding to each study is proportional to the sample size, and the horizontal line shows the corresponding 95% CI of the relative risk (RR) displayed on the right.

RETRACTED

#### Postoperative mortality

These five studies [10-14] also described the postoperative mortality of patients with pancreatic cancer. Since no between-study heterogeneity was observed (*P* = 0.597, I^2^ = 0.0%), a fixed effects model was used for analysis. No significant difference was identified in postoperative mortality between the PD/ELND group and the standard PD group according to the meta-analysis result (RR = 1.14, 95% CI 0.43 to approximately 3.00, *P* = 0.789, Figure 5).

**Figure 5:** **Forest plot for the postoperative mortality between the pancreatoduodenectomy with extended lymphadenectomy (PD/ELND) group and the standard pancreatoduodenectomy (PD) group.** The size of the black box corresponding to each study is proportional to the sample size, and the horizontal line shows the corresponding 95% CI of the relative risk (RR) displayed on the right.

#### Operative time

In these five studies [10-14], the operative time of pancreatic cancer patients with different operations was included. A random effects model was adopted because significant between-study heterogeneity was shown in this analysis (*P* = 0.000, I^2^ = 99.9%). The operative time of the PD/ELND group was significantly longer than that of the standard PD group according to the analysis (WMD = −1.03, 95% CI −1.96 to approximately −0.10, *P* = 0.029, Figure 6).

**Figure 6:** **Forest plot for the operative time between the pancreatoduodenectomy with extended lymphadenectomy (PD/ELND) group and the standard pancreatoduodenectomy (PD) group.** The size of the black box corresponding to each study is proportional to the sample size, and the horizontal line shows the corresponding 95% CI of the relative risk (RR) displayed on the right.

#### Amount of blood transfusions

There were four studies [10,12-14] that provided the amount (in volume) of blood transfusions. As between-study heterogeneity existed (*P* = 0.000, I^2^ = 98.8%), a random effects model was used for analysis. No significant difference was observed between the PD/ELND group and the standard PD group (WMD = −0.14, 95% CI −0.36 to approximately 0.08, *P* = 0.213, Figure 7).

**Figure 7:** **Forest plot for the amount of blood transfusions between the pancreatoduodenectomy with extended lymphadenectomy (PD/ELND) group and the standard pancreatoduodenectomy PD group.** The size of the black box corresponding to each study is proportional to the sample size, and the horizontal line shows the corresponding 95% CI of the relative risk (RR) displayed on the right.

RETRACTED

#### Hospital stay

Finally, the hospital stays days of pancreatic cancer patients after two different operations were reported in these five studies [10-14]. Because between-study heterogeneity existed (*P* = 0.000, I^2^ = 99.6%), a random effects model was adopted for analysis. No significant difference was observed in hospital stays between the PD/ELND group and the standard PD group (WMD = −0.32, 95% CI −2.57 to approximately 1.94, *P* = 0.784, Figure 8).

**Figure 8:** **Forest plot for hospital stays between the pancreatoduodenectomy with extended lymphadenectomy (PD/ELND) group and the standard pancreatoduodenectomy (PD) group.** The size of the black box corresponding to each study is proportional to the sample size, and the horizontal line shows the corresponding 95% CI of the relative risk (RR) displayed on the right.

## Discussion

The advantage of PD/ELND over standard PD for the treatment of pancreatic cancer is still controversial. To provent the lymphatic metastasis of pancreatic cancer, a PD/ELND, which extends the surgical region, makes sense to avoid recurrence. However, according to several studies, the results were not consistent. Although PD/ELND significantly increased the resection rate, it might fail to correspondingly improve the survival time for patients. In addition, PD/ELND could bring more complications, which subsequently eroded postoperative quality of life and raised mortality [15-17].

This meta-analysis showed that PD/ELND resulted in a significantly lower 3-year survival rate, but prolonged operative time and resulted in a higher incidence of postoperative complications for patients with pancreatic cancer compared with standard PD. Additionally, no significant difference was observed in 1- or 5-year survival rate, postoperative mortality, hospital stay and the volume of blood transfusions between the two groups.

Many meta-analyses were performed with extended lymphadenectomy for other malignancies, such as breast cancer [18,19] and papillary thyroid carcinoma [20,21]. The conclusions were various, and the evidences of the clinical improvements were rather weak. Authors stressed that more RCTs are needed for further understanding the feasibility of extended lymphadenectomy, which was also appropriate for pancreatic cancer.

Studies included in this meta-analysis came from different countries with various ethnic groups. The random allocation method was applied in each study, and the basic characteristics for patients from the test group and control group were not different, all of which guaranteed the representativeness of the conclusion. However, there were some limitations that need to be noted. The number of RCTs and cases contained in this evaluation were rather small. Moreover, variance also existed in the method of blinding, lymph node dissection, comprehensive treatment program after surgery and in postoperative follow-up time. All of these factors affected the strength of evidences and comprehensiveness of this systematic evaluation. Therefore, more prospective RCTs with large sample sizes and adequate follow-up times are necessary to verify the efficacy of PD/ELND for treatment of pancreatic cancer.

RETRACTED

## Conclusions

Based upon the above statistical results, we conclude that PD/ELND fails to gain advantages over standard PD in the survival rate of patients with pancreatic cancer, but may increase the operative time and the incidence of postoperative complications.

### Consent

Written informed consent was obtained from the patient for the publication of this report and any accompanying images.

## Abbreviations

CI: Confidence interval; ELND: Extended lymphadenectomy; PD: Pancreatoduodenectomy; PD/ELDN: Pancreatoduodenectomy with extended lymphadenectomy; RCT: Randomized controlled trial; RR: Relative risk; WMD: Weighted mean distance.

## Competing interests

The authors declare that they have no competing interests.

## Authors’ contributions

XBX collected material, carried out statistical analysis and wrote the manuscript; HZ provided evaluating data; PZ help to complete the article; LC was involved in editing the manuscript and statistical analysis; all authors provided final approval to the submitted version of the article.
